This article has been retracted.

# mir-204-5p Acts as a Tumor Suppressor by Targeting DNM2 in Osteosarcoma Cells

**DOI:** 10.1155/2022/8944588

**Published:** 2022-02-09

**Authors:** Liangliang Qu, Zhongqiu Li, Pinduan Liu

**Affiliations:** ^1^Department of Orthopedics, The First Affiliated Hospital of Jinzhou Medical University, Jinzhou 121001, Liaoning, China; ^2^Department of Hepatobiliary Diseases, The First Affiliated Hospital of Jinzhou Medical University, Jinzhou 121001, Liaoning, China

## Abstract

Osteosarcoma is a malignant bone tumor composed of interstitial cells. We aim to seek the function of mir-204-5p/DNM2 in osteosarcoma cells. From April 2017 to August 2019, 58 cases of cancer tissues and paracancer tissues were obtained from patients with osteosarcoma in our hospital. qPCR was used to detect mir-204-5p in excisional cancer tissues and paracarcinoma tissues of osteosarcoma patients. The overexpression vector of mir-204-5p was established and transfected into osteosarcoma cells, and the propagation, invasiveness, migration, and apoptosis of osteosarcoma cells were observed. StarBase was employed to forecast the binding site of mir-204-5p and DNM2. The targeting connection of mir-204-5p with DNM2 was detected via double luciferase reporter gene. mir-204-5p was lessened in osteosarcoma (*p* < 0.05). mir-204-5p overexpression suppressed propagation and accelerated apoptosis of osteosarcoma cells (*p* < 0.05). The results of double luciferase reporter gene revealed that the fluorescence activity of mir-204-5p was obviously declined when binding to DNM2 (*p* < 0.05). mir-204-5p functions as a tumor inhibitor by targeting DNM2 in osteosarcoma cells. Our research is helpful to provide new ideas for clinical treatment.

## 1. Introduction

Osteosarcoma is a malignant bone tumor composed of interstitial cells, which often develops in children and adolescents and produces osteoid and immature bone [1, 2]. At present, the treatment of osteosarcoma includes surgical resection combined with systemic chemotherapy to control micrometastasis. For patients with local osteosarcoma, this will result in about 70% of 5-year event-free survival, while the overall survival rate of patients with metastatic or recrudescent diseases is <20% [3, 4]. Although there are many attempts to enhance the treatment by increasing the dose and adding chemotherapeutic agents in large clinical trials, the survival rate of osteosarcoma has been stagnant in the past three decades [5]. Therefore, it is necessary to find new effective treatment methods.

MicroRNA (miRNA) is a small RNA molecule, which plays a role in gene silencing and translation inhibition by binding with target mRNA [6, 7]. More and more evidences have shown that many physiological processes and pathological results (including cancer) are highly dependent on miRNA [8]. miRNA-based therapy has great potential to restore or inhibit miRNA expression and activity, which can be used as a negative modulator of gene expression and regulate a series of biological functions, including cell survival, proliferation, apoptosis, tumor growth, and metastasis [9]. As a member of miRNA family, the pathological function of mir-204-5p (mir-204) has been observed in some diseases including pulmonary hypertension, diabetes, and various types of cancers [7]. Some studies have shown that mir-204 decreased in KGN cells and ovarian cortex tissues of patients with polycystic ovary syndrome [10]. It has also been studied that downregulation of miR-204 in smooth muscle of pulmonary arterioles may be related to pulmonary hypertension [11]. All these reveal that the imbalance of mir-204-5p may be bound up with the development of diseases. The miR-204-5p is abnormal in many diseases. Previous research has shown that miR-204-5p in glioma tissue is obviously lower than that in normal brain tissue, and miR-204-5p is obviously bound up with the grade of glioma [12]. Other researchers have shown that miR-204-5p in prostate carcinoma tissues and serum samples with osseous metastasis is lower than that in prostate cancer tissues and serum samples without osseous metastasis, which is related to the late clinicopathological features of prostate carcinoma patients and the presence or absence of poor bone metastasis [13].

Nevertheless, miR-204-5p in osteosarcoma is still unclear. Therefore, in this research, the expression and influence of mir-204-5p in osteosarcoma were investigated to provide new ideas for clinical treatment.

## 2. Materials and Methods

### 2.1. Specimen Collection

Recent reports indicate that abnormal overexpression of DNM2 protein can lead to dysfunction of internal circulation, resulting in unbalanced expression of regulatory growth factor receptor (including epidermal growth factor receptor) on the cells surface, thus accelerating the growth, invasiveness, and proliferation of abnormal cells [14]. Studies have also shown that NME2 plays a part in regulating the movements and metastases of tumor cells [15, 16]. From April 2017 to August 2019, 58 cases of carcinoma tissues and corresponding adjacent normal tissues were obtained from sufferers with osteosarcoma in our hospital, including 34 males and 24 females. The average age was 17.82 ± 4.23 years old. The average weight was 55.57 ± 4.89 kg.

### 2.2. Exclusion and Inclusion Criteria

  Inclusion criteria: all patients were confirmed as having osteosarcoma by MRI or CT [17]. This research was ratified by the ethics committee of our hospital, and the family members and patients were notified and signed the informed consent before the experiment.
  Exclusion criteria: patients with severe hepatic and renal insufficiency, patients who had received other treatments before the experiment, and patients who were mentally disturbed and uncooperative.

### 2.3. Main Instruments and Materials

There was osteosarcoma cell U-2 OS (Shanghai Xuanya Biotechnology Co., Ltd.), real-time fluorescence quantitative PCR instrument (Guangzhou Huafeng Biotechnology Co., Ltd.), 10% fetal bovine serum (Shanghai Lianshuo Baowei Biotechnology Co., Ltd.), DMEM medium (Qingdao Jieshikang Biotechnology Co., Ltd.), transfection reagent Lipofectamine™ 2000 (Suzhou Yuheng Biotechnology Co., Ltd.), apoptosis kit (Hangzhou Beiwo Medical Technology Co., Ltd.), TRIzol reagent (Beijing Biolab Technology Co., Ltd.), CCK8 kit (Beijing Jinkong Biotechnology Co., Ltd.), UV spectrophotometer (Shanghai Qinxiang Scientific Instrument Co., Ltd.), BD flow cytometer (Beijing Delika Biotechnology Co., Ltd.), transwell chamber (Shanghai Shengbo Biomedical Technology Co., Ltd.), reverse transcriptase (Shanghai Kanglang Biotechnology Co., Ltd.), enzyme-labeling instrument (Beijing Image Trading Co., Ltd.), and synthesis of mir-204-5P and internal reference primers (Beijing Zhongmei Taihe Biotechnology Co., Ltd.) (Table 1).

### 2.4. Methods

#### 2.4.1. Determination of mir-204-5p via qPCR

The mir-204-5p in osteosarcoma and adjacent tissues was tested via qRT-PCR, and the general RNA was obtained from the specimen by TRIzol in strict accordance with operation specifications. The level and purity of general RNA were tested by the ultraviolet spectrophotometer. RNA with OD260/OD280 ratio of 1.8 with 2.0 was obtained, and then, cDNA was compounded by reverse transcriptase and oligonucleotide according to the operating instructions. The transcription reaction system (20 *μ*L) consists of buffer (4 *μ*L), reverse transcriptase (2 *μ*L), total RNA (2 *μ*L), and RNase-free water (12 *μ*L). Reaction conditions were at the waterbath at 42°C for 1 hour and waterbath at 95°C for 5 minutes. PCR was used for amplification reaction. U6 was used as internal reference, and the specific primers of mir-204-5p were used to detect the mir-204-5p in fluorescence quantitative PCR according to the operation instructions. The PCR reaction system (20 *μ*L) consists the following: forward primer (0.4 *μ*L), reverse primer (0.4 *μ*L), and 0.5 *μ*L of Taq DNA polymerase, and the rest was supplemented with ddH_2_O. The reaction conditions were predenatured at 95°C for 30 s, at 95°C for 5 s, and at 60°C for 30 s, with a total of 40 cycles. Three multiple holes were set in each experiment, and the experiment was repeated three times. The experimental results were analyzed by the relative quantitative method, and the relative expression of mir-204-5p was calculated by 2^−△△CT^.

#### 2.4.2. Cell Culture and Transfection

The high-sugar DMEM medium containing 10% fetal bovine serum solution + 1% penicillin/streptomycin solution was used for routine subculture. The growth conditions were in a cell incubator at 37°C with 5% carbon dioxide, and the cells were inoculated in a 6-hole plate, so that the cell density reached 60–70%. The cells were treated with miR-204-5pmimcs and NC mimics vectors through the Lipofectamine™ 2000 kit according to the operation instructions.

#### 2.4.3. Detection of Cell Growth Curve

The transfected cells were made into suspension, which was inoculated into 96-hole plates with 100 *μ*L/well of cell suspension, respectively, and each well was provided with three multiple wells. At four time points (24 h, 48 h, 72 h, and 96 h), 20 *μ*L of cell proliferation colorimetric assay reagent (cck8) was added to each well at 2 h before the end of culture and then cultivated at 37°C and 5%CO_2_. After 2 h, the absorbance was measured at 490 nm by using an automatic enzyme-labeling instrument to observe the cell proliferation. The experiment was reduplicated three times.

#### 2.4.4. Detection of the Migratory and Invasive Ability of Cells

The cell suspension (5 × 10 ^4^ cells/hole) was put in the upper compartment in serum-free culture media. The media comprising 10% FBS in the lower compartment were used as a chemic attractant. After culture for 24 hours, cells that did not migrate were removed from the upper surface of the filter by scrubbing with cotton swabs. Next, the film was fixed with 4% formaldehyde at ambient temperature for 15 minutes and dyed with 0.5% crystal violet for 15 minutes. For the determination of cell invasion, 8% matrix glue was applied in the above steps. The experiment was reduplicated three times.

#### 2.4.5. Apoptosis Detection

The apoptosis detection kit was used to detect the apoptosis of cells, and the test followed the operation instructions. The BD flow cytometer was used to detect the cells which had been transfected for 48 hours and stained by Annexin V and PI in a 6-hole plate, and the experiment was repeated three times.

#### 2.4.6. Detection of the Targeting Connection of mir-204-5p with DNM2 by Double Luciferase

A DNA fragment of DNM2mRNA 3′-UTR comprising the putative combining site of mir-204-5p was synthesized. Then, the fragment was subcloned to Xho I and Not I sites downstream of the coding region of renilla luciferase in psiCHECK2 vector and verified by Sangon Biotech sequencing. PsiCHECK2-DNM2-wt or PsiCHECK2-DNM2-mut was constructed, and miR-204-5pmimcs or miR-NC and Wt-DNM2 or Mut-DNM2 were transfected into cells by Lipofectamine™ 2000. After transfection for 48 hours, cells were obtained. Next, the activities of firefly and Ranilla luciferase were analyzed by double luciferase reporting assay (Promega) in line with the makers' specifications.

### 2.5. Statistical Analysis

The differences were verified by statistic software SPSS 21.0 (SPSS, Inc., Chicago, IL, USA). The *t*-test was applied to express the measurement data, which were expressed by the mean number ± standard deviation (*x* ± sd). Repetitive measurement and analysis of variance were used to compare multiple time points within the group, which was expressed by F. The difference was statistically significant with *p* < 0.05.

## 3. Research Findings

### 3.1. mir-204-5p in Osteosarcoma and Adjacent Tissues

The relative expressions of mir-204-5p in osteosarcoma and adjacent tissues were (1.21 ± 0.53) and (3.14 ± 0.86), respectively. Compared with that in paracarcinoma tissues, the relative expression level of mir-204-5p in osteosarcoma tissue was lower (*p* < 0.05) (Figure 1).

### 3.2. Effect of mir-204-5p after Transfection

After transfection, the mir-204-5p in mir-204-5pmimcs and NC mimics was (2.69 ± 0.62) and (1.27 ± 0.56), respectively. Compared with that in NC mimics, the relative expression of mir-204-5p in mir-204-5pmimcs was higher after transfection (*p* < 0.05), indicating that the expression of mir-204-5p was obviously upregulated (Figure 2).

### 3.3. Growth of Osteosarcoma Cells after Transfection

At 24 h, there were no differences in the development of osteosarcoma cells between mir-204-5pmimcs and NC mimics (*p* > 0.05). From 48 h to 96 h, the growth of osteosarcoma cells of mir-204-5pmimcs was obviously lower compared with that of NC mimics (*p* < 0.05), which indicated that the growth of osteosarcoma cells was inhibited when mir-204-5p was obviously enhanced (Figure 3).

### 3.4. Migration and Invasiveness of Osteosarcoma Cells after Transfection

After transfection, the number of cell migration of mir-204-5pmimcs and NC mimics was (75.18 ± 5.49) and (116.54 ± 9.41), respectively. Compared with that of NC mimics, the number of cell migration of mir-204-5pmimcs was lower (*p* < 0.05) (Figure 4). After transfection, the number of cell invasion of mir-204-5pmimcs and NC mimics was (61.42 ± 5.75) and (104.46 ± 8.19), respectively. Compared with that of NC mimics, the number of cell invasion of mir-204-5pmimcs was lower (*p* < 0.05) (Figure 5).

### 3.5. Apoptosis of Osteosarcoma Cells after Transfection

After transfection, the apoptotic rates of mir-204-5pmimcs and NC mimics were (32.41 ± 3.82)% and (5.71 ± 1.59)%, respectively. The apoptotic rate of mir-204-5pmimcs was higher than that of NC mimics (*p* < 0.05) (Figure 6).

### 3.6. mir-204-5p Targeted DNM2 Directly

We forecasted the binding locus of mir-204-5p with DNM2 by StarBase, and the findings of double luciferase reporter gene revealed that mir-204-5pmimcs could reduce the luciferase activity of DNM2-Wt, but it did not impact the luciferase activity of DNM2-Mut, indicating that the fluorescence activity of mir-204-5pmimcs decreased significantly when binding to DNM2 (*p* < 0.05) (Figure 7). Then, we observed the effect of interfering DNM2 on osteosarcoma cells and reexpressed DNM2 in osteosarcoma cells treated with mir-204-5p. The findings revealed that DNM2 reexpression saved the growth defects after transfection of a mimetic agent (Figure 8).

## 4. Discussion

Similarly, research studies have shown that miR-204-5p in cells and patients with esophageal squamous cell carcinoma is lower than that in normal tissues and cells, and it has also shown that the continuous decline of miR-204-5p is bound up with unfavorable prognosis of sufferers [18].

In this experiment, we first tested mir-204-5p in osteosarcoma and paracarcinoma tissues by qRT-PCR. The findings revealed that mir-204-5p in osteosarcoma tissue was lower than that in adjacent tissues. The findings indicated that mir-204-5p was declined in osteosarcoma, and it might be a carcinogen in osteosarcoma. More and more evidences have shown that miRNA can be used as a cancer suppressor or oncogene to interfere with the progress of cancer [19]. We observed the influence of mir-204-5p on the biological behavior of osteosarcoma cells by interfering with miR-204-5P in osteosarcoma cells. The findings revealed that upregulation of mir-204-5p obviously inhibited the growth activity and migrating of osteosarcoma cells and accelerated apoptosis. The research has shown that miR-204-5p has been previously declined in melanoma compared with melanocytic nevus, and miR-204-5p mimetic can lead to the reduction of melanoma cell growth and continued migration and invasion of tissues [20]. Other research studies have revealed that miR-204-5p is significantly downregulated in triple negative breast carcinoma, and miR-204-5p ectopic expression in breast carcinoma cells can greatly reduce the migratory and invasiveness of carcinoma cells [21]. Other research studies have shown that mir-204-5p overexpression in human hepatocellular carcinoma cell strains can inhibit the viability of cells and increase apoptosis [22]. All these indicate that the biological behavior of tumor cells can be influenced by regulating miR-204-5p. DNM2 is a GTP enzyme, which plays a crucial role in the formation and transportation of intracellular vesicles, cytokinesis, and receptor endocytosis [23, 24]. However, there is no specific clinical study on the role of the two in osteosarcoma. In this research, we predicted the binding locus between mir-204-5p and DNM2 through StarBase, and the results of double luciferase reporter gene indicated that the fluorescence activity of mir-204-5pmimcs decreased obviously when binding to DNM2. Then, we observed the effect of interfering DNM2 on osteosarcoma cells and reexpressed DNM2 in osteosarcoma cells treated with mir-204-5p.

## 5. Conclusion

In conclusion, mir-204-5p is declined in osteosarcoma, and its upregulation can effectively inhibit growth activity of cell and induce apoptosis, and mir-204-5p may act on osteosarcoma cells by directly targeting DNM2. The findings revealed that DNM2 reexpression saved the growth defects after transfection of a mimetic agent. These findings revealed that mir-204-5p might control the biological behavior of osteosarcoma cells by directly targeting DNM2.

## Figures and Tables

**Figure 1:** Relative expression of mir-204-5p in osteosarcoma and adjacent tissues. ^*∗*^Comparison with the adjacent tissues (*p* < 0.05).

**Figure 2:** Effect of mir-204-5p after transfection. ^*∗*^Comparison with NC mimics (*p* < 0.05).

**Figure 3:** Growth of osteosarcoma cells after transfection. ^*∗*^Comparison with NC mimics (*p* < 0.05).

**Figure 4:** Migration of osteosarcoma cells after transfection. ^*∗*^Comparison with NC mimics (*p* < 0.05).

**Figure 5:** Invasion of osteosarcoma cells after transfection. The number of cell invasion of mir-204-5pmimcs was lower than that of NC mimics (*p* < 0.05). ^*∗*^Comparison with NC mimics (*p* < 0.05).

**Figure 6:** Apoptosis of osteosarcoma cells after transfection. ^*∗*^Comparison with NC mimics (*p* < 0.05).

**Figure 7:** mir-204-5p targeted DNM2 directly. (a) Target gene map. (b) Results of double luciferase reporter gene: mir-204-5pmimcs could reduce the luciferase activity of DNM2-Wt, but it had no effect on the luciferase activity of DNM2-Mut (*p* < 0.05). ^*∗*^Comparison with NC mimics (*p* < 0.05).

**Figure 8:** Rescue experiment chart. The reexpression of DNM2 saved the growth defects, migration, and invasion after transfection of mimetic agents. (a) Growth of cells in each group after retransfection of DNM2. (b) Migration of cells in each group after retransfection of DNM2. (c) Invasion of cells in each group after retransfection of DNM2. (d) Apoptosis in each group after retransfection of DNM2. ^*∗*^Comparison with NC mimics (*p* < 0.05).

**Table 1:** Primers sequence.

	Forward primers (5′-3′)	Reverse primers (5′-3′)
miR-204-5p	GCCAGATCTGGAAGAAGATGGTGGTTAGT	GGCGAATTCACAGTTGCCTACAGTATTCA
U6	CTCGCTTCGGCAGCACA	AACGCTTCACGAATTTGCGT

## Data Availability

The datasets used and/or analyzed during the current study are available from the corresponding author upon request.
